# Infectious clone construction and pathogenicity confirmation of Cotton leaf curl Multan virus (CLCuMuV), Ramie mosaic virus (RamV) and Corchorus yellow vein Vietnam virus (CoYVV) by southern blot analysis

This article has been retracted.

**DOI:** 10.1371/journal.pone.0251232

**Published:** 2021-05-14

**Authors:** Muhammad Arif, Saif ul Islam, Saqer S. Alotaibi, Ahmed M. Elshehawi, Mohamed A. A. Ahmed, Abdullah M. Al-Sadi

**Affiliations:** 1 Department of Plant Protection, Fujian Agriculture and Forestry University, Fuzhou, China; 2 Vegetable Research Institute, Guangdong Academy of Agricultural Sciences, Guangzhou, China; 3 Department of Biotechnology, College of Science, Taif University, Taif, Saudi Arabia; 4 Plant Production Department (Horticulture—Medicinal and Aromatic Plants), Faculty of Agriculture (Saba Basha), Alexandria University, Alexandria, Egypt; 5 Department of Plant Sciences, College of Agricultural and Marine sciences, Sultan Qaboos University, Alkhound, Oman; Harran Üniversitesi: Harran Universitesi, TURKEY

## Abstract

Geminiviruses are insect-transmissible, economically vital group of plant viruses, which cause significant losses to crop production and ornamental plants across the world. During this study, infectious clones of three devastating begomoviruses, i.e., *Cotton leaf curl Multan virus* (CLCuMuV), *Ramie mosaic virus* (RamV) and *Corchorus yellow vein Vietnam virus* (CoYVV) were constructed by following novel protocol. All infectious clones were confirmed by cloning and sequencing. All of the infectious clones were agro-inoculated in Agrobacterium. After the agro-infiltrations, all clones were injected into *Nicotiana benthamiana* and jute plants under controlled condition. After 28 days of inoculation, plants exhibited typical symptoms of their corresponding viruses. All the symptomatic and asymptomatic leaves were collected from inoculated plants for further analysis. The southern blot analysis was used to confirm the infection of studied begomoviruses. At the end, all the products were sequenced and analyzed.

## Introduction

Begomoviruses, belonging to the largest family of plant viruses (*Geminiviridae*) have ssDNA molecule enclosed in twinned particles and transmitted with the help of haplotype insect vector haplotype whitefly (*Bemisia tabaci*) to dicotyledonous plants. Begomoviruses are further divided into two types, i.e., monopartite having only DNA A genome of 2.7 kb size, while bipartite contain both DNA A and DNA B genomes of 2.5–2.7 kb size [1–3]. The DNA A component of bipartite is implied in virions production and replications, but need DNA B for systemic infection, host range determination, symptoms expression and nuclear localization [4, 5]. Both DNA A and DNA B components contain a non-coding region with ~200 bp sequence which holds the sequence motifs required for the determination, replication and gene expression [6, 7].

The cloning of a full-length begomovirus genome is normally completed directly from isolated dsDNA [8, 9] by PCR amplicon of whole genome [10] or from RCA generated genome component [11–13]. The co-infection of viruses of two different *geminivirida*e genera has an obligation of intergenic recombination. Genetic recombination directs not only to diversity of host genome, but also to extend it in previous diversity, which was held in virus genome. It provides new paths for evolution of virus and co-evolution of begomoviruses that may leads to new prospects for understanding the complexity of begomoviruses [14]. The co-infection of begomovirus with dicot-infecting master virus within the same host is common nowadays and three cases have been reported [15]. From these cases, every time host plant was different with member of different plant families [15–17] described the co-infection of master-begomovirus (*Chickpea chlorotic dwarf virus;* CPCDV) in weed, cotton and squash with different families, i.e., Asteraceae, Malvaceae and Cucerbitaceae, respectively.

Normal infectious clone construction depends on cloning of a full-length genome, which is subsequently sub-cloned as a tandem, one and half or two genomes components into suitable vector for agro-inoculation. The construction of genome components comprising two replication origins is a slow and lengthy process [18]. In some situations excised unit length cloned DNA bearing single copies of virus genome act as an infectious clone of certain plant viruses [19–21]. Previous studies had described that most infectious clones entail tandem repeat constructs of geminivirus/begomovirus genomes to extend their pathogenicity [22–25], which makes cloning procedure more complex. The process make multimeric constructs of begomoviruses for tickly selection and design of cloning sites, pursued by aggregation of viral genomic fragments yielded by restriction endonucleases has become an exhausting phenomenon [26, 27]. Furthermore, perfectness of inserts should be checked carefully to choose the clones, which have tandem-repeat viral genomes. Recently a fresh technique rolling circle amplification (RCA) has been established for linear or symmetrical amplification of targeted DNA or betasatellites [28]. Multimeric infectious clones of several geminiviruses were yielded with the help of RCA [29, 30].

The *cotton leaf curl disease* (CLCuD) is caused by complex of begomoviruses, including *cotton leaf curl Multan virus* (CLCuMuV) with its disease specific *betasatellite cotton leaf curl Multan betasatellite* (CLCuMuB) in many south Asian countries, including Pakistan, China and India. The CLCuMuV is one of the causal agent of CLCuD, which devastated the cotton industry of Pakistan during 1990s had recently established in southern China by infecting *Rosa sinensis* and many other host plants [31]. During 2015, some jute plants showing typical viral symptoms were observed in China. The observed symptoms on infected plants were vein yellowing, leaf mosaic, and deformation. There was a huge population of whitefly feeding on these plants, which recommended the etiology of begomovirus. Isolation of DNA fragment, cloning and sequencing have confirmed it as *Corchorus yellow vein Vietnam virus* (CoYVV) [32].

Ramie (*Boehmeria nivea*) is regarded as most ancient and important fiber crop in many countries, including China and India. This plant is well recognized for its durable and strong natural fiber worldwide. It is a semi-perennial plant, produced in tropical and temperate regions. The *ramie mosaic virus* (RamV) was identified in 2010 in Zhejiang and Jiangsu provinces of China. Virus isolates having DNA A and DNA B from both provinces were detected and described. Soon after that it started to migrate from one place to another within the China [33, 34]. Due to less information about diseases and pests associated with ramie, it is difficult to index, identify and classification of ramie diseases. Here in this study, infectious clones of three begomoviruses CLCuMuV, CoYVV and RamV were constructed and agro-inoculated into *N*. *benthamiana* for determine their pathogenicity and molecular studies.

## Materials and methods

### Collection of samples and DNA extraction

In this study, three begomoviruses, i.e., CLCuMuV, CoYVV and RamV were used. The viruses were collected from different locations in Fujian province, China. The CLCuMuV was detected from infecting plants of *H*. *sabdariffa* and *H*. *esculentus*. Disease incidence was high with huge population of whitefly (*B*. *tabaci*) cryptic species on infected plants. Full length DNA A and DNA B were detected from infected plants that were further cloned and sequenced. The CoYVV was found infecting jute plants in different locations of Fujian province. Full length CoYVV DNA A and DNA B obtained from PCR products were cloned and sequenced. RamV was found infecting ramie plants in Fujian province. RamV DNA A and DNA B were obtained from PCR products, cloned and sequenced. Nucleotide sequence identity of all these begomoviruses was checked by using the BLASTn.

### Construction of infectious clone and *Agrobacterium* infiltration

For infection of all begomoviruses with *N*. *benthamiana* strain EHA105 having plasmid of interest was developed at an optical density of 600 nm (OD600) at 28°C on liquid broth medium added with two antibiotics kanamycin (50ug/ul) and rifampicin (50ug/ul). All cultures were centrifuged at 12000 RPM (g) for 1-minute and followed by resuspension method with an induction medium [10 mM 2-(N-morpholino) ethane sulfonic acid (MES), pH 5.6, 10 mM MgCl2 and 150 μ M Acetosyringne].

For the construction of infectious clones, RCA product was partially digested with SalI enzyme. Head to tail tandem repeat dimers was cloned by using SalI in pCAMBIA1301 binary vector (CAMBIA, Canberra, Australia). The illustration of an infectious clone is shown in Fig 1. Identification of these infectious clones was confirmed by sequencing. The identified sequences confirmed CLCuMuV, CoYVV and RamV infectious clones. The *Agrobacterium* strain GV3101 was transformed separately with the recombinant pCAMBIA1301 bearing tandem repeats. The culture of transformed *Agrobacterium* was allowed to grow about OD600 = 1.0 and then incubated in induction buffer 10 mM MgCl_2_, 100 mM MES (pH 5.7), 100 M Acetosyringne] for ~3 hours at room temperature. The *Agrobacterium* cultures of virus and satellite were mixed (1:1) before the agro-infection. The mixtures of induced cultures were in-filtered into abaxial part of cotyledon leaves of 2-week old seedlings. After *Agrobacterium* infiltration, *N*. *benthamiana* plants were retained in an incubator at 25°C with a relative humidity of 80%. After 20 days of *Agrobacterium* infiltration, plants were injected with infection clones of CLCuMuV, CoYVV and RamV [35]. CoYVV was also inoculated in jute from which it was identified. A needless syringe was used for injection in the lower lamina of young tobacco leaves. The agro-inoculated plants were maintained in a controlled chamber at 25°C [36]. After inoculation of all these viruses, *N*. *benthamiana* and jute plants were allowed to grow under standard greenhouse conditions (16 hours day length and 22–24°C temperature). The DNA and RNA were extracted from newly grown leaves of infected plants after 28 days of *Agrobacterium* infiltration. Total DNA and RNA were used to check the expression level of the target gene.

**Fig 1:** Illustration of construction of infectious clone of begomoviruses.

### Confirmation of infection by Southern Blot analysis

Southern blot analysis discloses the complete information of DNA abundance, identity and size. This technique is attractive because of differentiating DNA fragments on the basis of size through electrophoresis and then shifting them into a membrane, hybridizing with the tagged sequence-specific probe, rinsing and at the end detecting marked DNA bands. Southern blotting was executed by following the protocol of (Roche, DIG application program for filter hybridization). 10 μg genomic DNA obtained of CLCuMuV, RamV and CoYVV were digested with EcoR1 and then allowed to run on agarose gel for overnight. After modifying with buffer containing 0.5M NaOH and 1.5M NaCl. The DNA was shifted to a nylon membrane by applying the capillary transfer technique. The shifted DNA was crossly hyperlinked with ultraviolet rays and then hybridized by DIG-labelled DNA probe at 42°C for a period of 16 hours. In the end, the membrane was examined with anti-DIG antibody formerly as it was built up with the help of CPSD substrate [37]. The original uncropped blot images (S1–S3 Figs) are provided in supplementary materials.

### Cloning and sequence analysis

PCR products were purified by using a gel extraction kit (Fermentas) according to the manufacturer’s instructions and were cloned into the pTZ57R/T vector (Fermentas). The PCR products (without cloning), as well as cloned products were sequenced (Macrogen, Korea). Sequences were analyzed using the Lasergene software package (DNASTAR Inc.) [38]. Sequence similarity was performed by comparing the sequence of other Begomoviruses/betasatellite sequence in the database (http://www.ncbi.nlm.nih.gov/BLAST/). Open reading frame (ORF) were located by using the ORF finder (http://www.ncbi.nlm.nih.gov//gorf/gorf.html)).

## Results and discussion

In this study three begomoviruses *Cotton leaf curl Multan virus* (CLCuMuV), *Corchorus yellow vein Vietnam virus* (CoYVV) and *Ramie mosaic virus* (RamV) were used. Briefly, CLCuMuV, CoYVV and RamV were detected from infecting plants of *H*. *sabdariffa* and *H*. *esculentus*, Jute and Ramie from different locations of Fujian province. These viruses were already identified in this province but from different host plants. The incidence of these viruses was much high as compared to earlier reported. Full-length genomes were sequenced from a commercial company (Beijing Genomics Institute, BGI, Shenzhen, China). For the construction of infectious clones of begomovirus, RCA product of each virus was partially digested with SalI enzyme. All these reactions were performed just for confirmation with previous studies [22, 39].

After 4 weeks of agro-inoculation, we discovered mix-infection of desired begomoviruses in *N*. *benthamiana*, but symptoms appearing time varied for each of begomoviruses as shown in Fig 2. Total DNA and RNA was obtained from infected upper leaves of the *N*. *benthamiana* plants. The PCR/RT-PCR has confirmed the co-infection with begomoviruses.

**Fig 2:** Expression of symptoms in *Nicotiana benthamiana* inoculated with (A), CLCuMuV (B) CoYVV (C) RamV and Southern-blot analysis of inoculated *N*. *benthamiana* plants.

To check the infectivity of these infectious clones, all clones were inserted into *Agrobacterium tumefactions* through heat shock transformation procedure before the agro-inoculation into *N*. *benthamiana*. The quality and pathogenicity CLCuMuV, CoYVV and RamV infectious clones were checked by agro-inoculation [40]. Total number of inoculated plants with *N*. *benthamiana* for each begomovirus infectious clone were agro-inoculated at leaf petiole stage mechanically with *Agrobacterium tumefactions* having chimeric constructs (infectious clone) of all these begomoviruses.

Viral assemblage and symptoms appearance for each begomovirus infected plants was checked in every week of post-inoculation. After 7 days of post-inoculation, no symptoms were observed on *N*. *benthamiana* plants for each begomovirus (Table 1). After 14 days of post-inoculation, initial little begomovirus symptoms start to develop on *N*. *benthamiana* for every begomovirus, but not all plants showed visible symptoms. After viewing these symptoms, it was confirmed that infectious clones have infectivity power to cause the infection in host plants. After 21 days of post-inoculation, visible symptoms grew further and became somewhat like characteristic symptoms of begomoviruses. The CoYVV didn’t induce symptoms in *N*. *benthamiana*. That plants which had not showed symptoms after 15 days were same as like, means that plant condition was much same as natural growth. After 28 days of post inoculation, full characteristic symptoms of CLCuMuV, CoYVV and RamV were observed. There were no symptoms’ induction in *N*. *benthamiana* for CoYVV, but its characteristic symptoms were observed in jute. It was concluded that CoYVV didn’t co-infect with other hosts and this virus has fulfilled the Koch’s postulates. Symptoms expressed by CLCuMuV infectious clone were mottling, vein clearing and stunted growth. The 4 out of 4 plants had showed typical CLCuMuV symptoms in *N*. *benthamiana*. For RamV, typical symptoms were observed in 3 out of 5 plants (Table 1). Other two plants failed to produce symptoms. Symptoms exhibited by CoYVV in *N*. *benthamiana* were yellow peels on leaf lamina. Symptoms expressed after 28 days of post-inoculation are shown in Fig 2. The *N*. *benthamiana* plants after agro-inoculation exhibited same type of symptoms observed in the field.

**Table 1:** Infectious clone agro-inoculation in *N*. *benthamiana* and other hosts.

Plant/Constructs	No. of Infected/inoculated plants	Incubation time	Symptoms	Southern blot detection
*N*. *benthamiana*	2/5	15*-28^α^	VC, M, LR	+
CLCuMuV				
*N*. *benthamiana*	4/4	9*-28 ^α^	MY, MVC	+
RamV				
*N*. *benthamiana*, Jute	0/4, 4/4	28*-28 ^α^	Y, CL, Chs, VB	_
		10*-28 ^α^		+
CoYVV				

Here

* = days for first appearance of symptoms

α = days at which leaves were collected for detection, + = positive results,— = negative results, Symptoms: VC = vein clearing, M = mosaic, LR = leaf rolling, MY = mild yellowing, MVC = mild vein clearing, Y = yellowing, CL = curled leaved, Chs = Chlorosis, VB = vein banding

The plants showing begomovirus symptoms as well as healthy plants were collected for further analysis. DNA was extracted from the symptomatic and asymptomatic leaves by CTAB method [41]. For verification of the presence of CLCuMuV, CoYVV and RamV in agro-inoculated infected leaves, southern blot analysis was executed. Southern-blot analysis results confirmed the infectivity of infectious clones which induce the symptoms in *N*. *benthamiana*. The plants that didn’t show symptoms, their southern-blot analysis was negative, while all others were positive as shown in Fig 2. The infectious clones of CLCuMuV, CoYVV and RamV has successfully induced symptoms in *N*. *benthamiana* by agro-inoculation. All these begomoviruses were detected from Fujian province by PCR/RCA. The co-infection of viruses from two different genera happens very seldom; for example, CPCDV a master virus and *Cotton leaf curl Burewala virus* (CLCuBuV) with its betasatellite [42]. The infectivity of CoGMV Bangladesh isolate was sustained by agro-inoculation in Jute plants. The infectious clones DNA A and DNA B has induced CoGMV characteristic symptoms in jute [40]. The pathogenicity of CoYVV and CoGMV by microprojectile bombardment in tobacco culture was performed but mechanical transmission of yellow mosaic disease didn’t give results because of having gum and phenolic compounds in jute plants [43].

The direct use of RCA products for sequencing [44], for mechanical inoculation of geminiviruses or for particle bombardment [29] might be less complicated than construction of agro-infectious (dimeric) clones. However, direct sequencing of amplified DNA by PCR/RCA might give unreadable nucleotides in obtained sequence. Moreover, particle bombardment of RCA products obtained from DNA of infected plant will never accurate than its inoculum has pure isolate. It is still believed that agro-inoculation with specific construction of infectious clones have substantial advantage over usage of RCA products as inoculation material.

It is believed that agro-inoculation with specific infectious clones have substantial advantage to fulfill the Koch’s postulates. It can provide virus host interactions and quick recognition of gene functions. Until now, infectious clones of almost all DNA viruses have been described, but still some of them are difficult to construct. Southern blot analysis can disclose the complete information about DNA abundance and identity. This technique has become an attractive because of differentiating the DNA fragments based on size through electrophoresis.

The construction of genome components comprising of two replication origins is a slow process [18]. While in some situations excised unit length cloned DNA bearing single copies of virus genome act as an infectious clone of certain viruses [19, 20]. Previous studies had described that most infectious clones entailed the tandem repeat constructs of geminivirus/begomovirus genomes to extend their pathogenicity [22–24], which induces the cloning procedure more complex. This process to make the multimeric constructs of begomoviruses involves tickly selection and design of cloning sites, pursued by aggregation viral genomic fragments yielded by restriction endonucleases is an exhausting phenomenon [26, 27]. Furthermore, perfectness of inserts should be checked carefully to choose clones, which have tandem-repeat viral genomes. Recently a fresh technique rolling circle amplification (RCA) has been established for linear or symmetrical amplification of targeted DNA or betasatellites [28]. The multimeric infectious clones of several geminiviruses were yielded with the help of RCA [29, 30]. The pathogenicity of CoYVV and CoGMV by micro projectile bombardment in tobacco culture was performed but mechanical transmission of yellow mosaic disease didn’t give results because of having gum and phenolic compounds in jute plants [43].

## Conclusion

Infectious clone of freshly identified CLCuMuV, CoYVV and RamV were constructed in this study. The CLCuMuV and RamV infectious clones significantly induced disease symptoms in *N*. *benthamiana* through agro-inoculation, while infectious clone of CoYVV didn’t induce symptoms in *N*. *benthamiana*; however, successfully induced symptoms in jute. It is concluded that CoYVV Fujian isolate is not capable to infect other hosts. Begomoviruses from different topographical locations can potentially interrelate with non-cognate betasatellites and alphasatellites with variegating deficiencies. Therefore, it is much possible that exchange of satellites may occur among begomoviruses. Like, CoYVV and CoGMV, which were identified in Vietnam but now causing severe infection throughout China. The CLCuMuV was a major constraint in India and Pakistan but now spreading in many malvaceous plants throughout China. The fundamental interaction between helper viruses and betasatellites is highly complex rather than already reported.

## Supporting information

S1 Fig Blot image of *Ramie mosaic virus* (RamV). (DOCX)

S2 Fig Blot image of *Corchorus yellow vein Vietnam virus* (CoYVV). (DOCX)

S3 Fig Blot image of *Cotton leaf curl Multan virus* (CLCuMuV). (DOCX)
